# A New Nonparametric Multivariate Control Scheme for Simultaneous Monitoring Changes in Location and Scale

**DOI:** 10.1155/2022/3385825

**Published:** 2022-07-04

**Authors:** Jin Yue, Liu Liu

**Affiliations:** ^1^College of Mathematics and Physics, Chengdu University of Technology, Chengdu 610059, China; ^2^School of Mathematics and VC & VR Key Lab of Sichuan Province, Sichuan Normal University, Chengdu 610068, China

## Abstract

Real-time monitoring of the breast cancer index is becoming increasingly important. It can help create advances in the diagnosis and treatment of breast cancer. In today's modern medical processes, simultaneously monitoring changes in observations in terms of location and scale are convenient for the implementation of control schemes but can be challenging. In this paper, we consider a new nonparametric control scheme for monitoring location and scale parameters in multivariate processes. The proposed method is easy to implement, and the performance of the proposed control procedure is discussed. Then, we compare the proposed scheme with some competing methods. Simulation results show that the proposed scheme can efficiently detect a range of shifts. The proposed chart can trigger an alert and timely discover the change of the breast cancer index.

## 1. Introduction

Control schemes play an important role in biosurveillance studies [1–9]. Control schemes have been frequently used for fault detection in quality control with products and health-care monitoring [10–14]. A process should be monitored using statistical means to determine whether a shift occurs, and action should be taken once the process is considered out-of-control (OC) [15–18]. Many researchers have discussed and proposed many useful charts, such as Shewhart charts [19, 20], cumulative sum (CUSUM) charts [21–30], and exponentially weighted moving average (EWMA) charts [31–38], to detect whether there is a change in quality characteristics in a process. These proposed control schemes can be used for data analysis, including control and forecasting, which are useful for fault diagnosis in practice. Most charts require that these observations be univariate and typically assume that these observations follow a normal distribution. Unfortunately, the assumption of multivariate normality is unrealistic in most cases and would lead to a poor performance if underlying assumptions are invalid.

Nonparametric control charts are important in manufacturing and service sectors when samples of observations are nonnormal. Some control schemes are used to monitor high-dimensional processes when we know little about the underlying distribution [39–42]. Most control schemes are designed to monitor location parameters. For example, Liu and Singh [43] introduced several multivariate rank tests based on data depth. Liu [44] used the concept of data depth to propose several new control charts to monitor multivariate process. Data depth provides an efficient metric of the process' performance without using parametric assumptions. In addition, Zou et al. [45] provided a multivariate spatial rank for monitoring high-dimensional processes with unknown parameters. For detecting the location changes in nonparametric multivariate processes, we also recommend the discussions by [46, 47]. To detect the changes in the location and scale of observations simultaneously, several monitoring methods are proposed in the literature, including Mukherjee and Chakraborti [48] and Chowdhury et al. [49]. Recently, Mukherjee and Marozzi [50] consider the sum of the squares of standardized Wilcoxon and the Bradley statistics for monitoring high-dimensional processes with unknown parameters which is advantageous in simultaneous monitoring of multiple aspects.

Recently, some schemes have been proposed to monitor the changes in location and scale simultaneously using a single chart. Performance advantages of these charts have been clearly established [51]. Lepage [52] discussed a nonparametric two-sample test for location and dispersion. Based on Lepage [52], Mukherjee and Marozzi [51] introduced new circular-grid charts for simultaneous monitoring of process location and process scale based on Lepage-type statistics. Meanwhile, Mukherjee and Marozzi [53] investigated a new single distribution-free Phase-II CUSUM procedure based on the Cucconi statistic for simultaneously monitoring changes in location and scale parameters of a process. In addition, Mukherjee and Sen [54] discussed a distribution-free (nonparametric) Shewhart-Lepage scheme for simultaneous monitoring of location and scale parameters using an adaptive strategy. Li et al. [55] and Shi et al. [56] provided powerful control schemes aimed at simultaneously monitoring the location and the scale parameters of any continuous process. Moreover, Zafar et al. [57] proposed a new parametric memory-type charting structure based on progressive mean under max statistic for the joint monitoring of location and dispersion parameters. Song et al. [58] introduced distribution-free adaptive Shewhart-Lepage-type schemes for simultaneous monitoring of location and scale parameters using information about symmetry and tail weights of the process distribution. Huang et al. [59] proposed a new statistical process monitoring scheme with a double-sampling plan for simultaneously monitoring location and scale shifts. Bai and Li [60] considered monitoring ordinal categorical factors for monitoring which considers shifts in the location or scale parameters of latent variables. For multivariate processes, Cheng and Shiau [61] proposed a distribution-free phase I monitoring scheme for both location and scale parameters based on the multisample Lepage statistic.

Although these literatures contain many control schemes for monitoring location and scale parameters simultaneously, much less focus has been placed on control strategies that simultaneously monitor location and scale parameters in multivariate processes. In this study, we propose a useful and easy-to-implement control scheme for simultaneously monitoring location and scale parameters, which is based on nonparametric location and scale hypothesis testing. Reference samples are denoted as phase I data streams, and test samples are denoted as phase II data streams. One problem is that the size of phase II increases with the number of data streams. Considering this issue, we performed hypothesis testing repeatedly with each new data stream. Thus, the amount of phase II data became a constant for each acquisition time.

The remainder of this paper is organized as follows: In Section 2, we review nonparametric hypothesis testing in detail. In Section 3, we propose a new scheme based on a hypothesis testing statistic for monitoring location and scale parameters. Then, we discuss the proposed method's performance and validity. In Section 4, we perform a simulation-based comparison to compare the proposed chart with other existing charts. In Section 5, breast cancer data are investigated to describe the performance of the proposed chart. Lastly, we briefly draw conclusions in Section 6.

## 2. Review of Nonparametric Hypothesis Testing

Hypothesis testing is a form of statistical inference that uses data from a sample to draw conclusions about a population parameter or a population probability distribution, considering reference sample {*X*_1,*t*_, *X*_2,*t*_, ⋯, *X*_*m*,*t*_} of size *m* and test sample {*Y*_1,*t*_, *Y*_2,*t*_, ⋯, *Y*_*n*,*t*_} of size *n*. Thus, null hypothesis *H*_0_ : *μ*_1_ = *μ*_2_, *σ*_1_^2^ = *σ*_2_^2^ versus alternative hypothesis *H*_1_ : *μ*_1_ ≠ *μ*_2_ or *σ*_1_^2^ ≠ *σ*_2_^2^, where *μ*_1_ is the location parameter of reference sample; *μ*_2_ is the location parameter of test sample; *σ*_1_^2^ and *σ*_2_^2^ are the scale parameters of the reference and test samples, respectively. We can use a reasonable statistical decision procedure to reject the null hypothesis *H*_0_. In real situations, it is difficult for us to identify the exact distribution of data streams. Therefore, nonparametric hypothesis testing is also introduced, which does not consider the distribution of the original data. For hypothesis testing about the location parameter, Mood [62] proposed the median test, which is based on the rank of each datum. Considering the interaction between the reference and test samples, Wilcoxon [63] and Mann and Whitney [64] introduced the Mann-Whitney-Wilcoxon statistic. In addition, rank-based nonparametric hypothesis testing of scale parameter is used in the literature [65–67].

### 2.1. Methods for Location Detection

In general, people often check whether there is a change for a given location parameter in a process. We often use the *t*-statistic under the assumption that the distribution is normal. However, there is a risk in using the *t*-statistic with unknown population distributions. Thus, some distribution-free statistics have been developed. Brown-Mood median testing is a useful nonparametric method. However, the bilateral test does not yield satisfactory results when *m* ≠ *n*. To use more information about the relative size of the reference sample and test sample, the Wilcoxon rank-sum test was developed. We assume that a reference sample of size *m* and test sample of size *n* are given, and we let *N* = *m* + *n*. Considering the pooled sample {*X*_1,*t*_, *X*_2,*t*_, ⋯, *X*_*m*,*t*_, *Y*_1,*t*_, *Y*_2,*t*_, ⋯, *Y*_*n*,*t*_} at time *t*, Mann and Whitney [64] developed the Mann-Whitney statistic as follows:

(1) $$\begin{array}{c} W_{1,t}=\overset{n}{\underset{j=1}{\sum }}\overset{m}{\underset{i=1}{\sum }}I\left\{X_{i,t}<Y_{j,t}\right\}. \end{array}$$

Therefore, the Wilcoxon rank-sum statistic is

(2) $$\begin{array}{c} W_{2,t}=W_{1,t}+\frac{n\left(n+1\right)}{2}, \end{array}$$

where *W*_2,*t*_ = ∑_*i*=1_^*n*^*R*_*i*,*t*_, and *R*_*i*,*t*_ is the rank of *Y*_*i*,*t*_ in the pooled sample {*X*_1,*t*_, *X*_2,*t*_, ⋯, *X*_*m*,*t*_, *Y*_1,*t*_, *Y*_2,*t*_, ⋯, *Y*_*n*,*t*_}. *E*(*W*_2,*t*_|*H*_0_) = *n*(*N* + 1)/2. It can be seen that [68]

(3) $$\begin{array}{c} E\left(W_{1,t}\left|H_{0}\right.\right)=\frac{mn}{2},\\ \text{Var}\left(W_{1,t}\left|H_{0}\right.\right)=\frac{mn\left(N+1\right)}{12}. \end{array}$$

Under the null hypothesis, we also calculate the approximate normal statistic when the sample *N* is sufficiently large.

### 2.2. Methods for Scale Detecting

A location parameter typically describes the position of a distribution, and a scale parameter is also an important characteristic that describes a distribution. When the distribution of observations is unknown, some distribution-free methods are typically used. Given a two-phase independent sample {*X*_1,*t*_, *X*_2,*t*_, ⋯, *X*_*m*,*t*_} ~ *F*(*μ*_1_, *σ*_1_^2^) and {*Y*_1,*t*_, *Y*_2,*t*_, ⋯, *Y*_*n*,*t*_} ~ *F*(*μ*_2_, *σ*_2_^2^). We assume that the location parameters of the two samples are equal (*μ*_1_ = *μ*_2_). Based on the Mann-Whitney statistic, Siegel and Tukey [65] proposed the Siegel-Tukey statistic. The implementation design of this statistic consists of the following steps: (1) mix the two samples {*X*_1,*t*_, *X*_2,*t*_, ⋯, *X*_*m*,*t*_, *Y*_1,*t*_, *Y*_2,*t*_, ⋯, *Y*_*n*,*t*_} in ascending order, *Q*_(1),*t*_, *Q*_(2),*t*_, ⋯, *Q*_(*m* + *n*),*t*_; (2) assign the rank *R*_*i*,*t*_′ of *Q*_(1),*t*_, *Q*_(2),*t*_, ⋯, *Q*_(*m* + *n*),*t*_ as shown in Table 1; and (3) calculate the *S*_*t*_ = ∑_*i*=1_^*n*^(*R*_*i*,*t*_′ − *n*(*n* + 1)/2); *R*_*i*,*t*_′ represents the rank of *Y*_*i*,*t*_.

Mood [62] also provided a useful test statistic for scale parameters. As before, we consider two sequences of {*X*_1,*t*_, *X*_2,*t*_, ⋯, *X*_*m*,*t*_} ~ *G*(*μ*_1_, *σ*_1_^2^) and {*Y*_1,*t*_, *Y*_2,*t*_, ⋯, *Y*_*n*,*t*_} ~ *G*(*μ*_2_, *σ*_2_^2^), where *μ*_1_ = *μ*_2_. The Mood statistic can be described as follows:

(4) $$\begin{array}{c} \text{M}{\text{D}}_{t}=\overset{n}{\underset{i=1}{\sum }}{\left(R_{i,t}-E\left(R_{i,t}\right)\right)}^{2}, \end{array}$$

where *R*_*i*,*t*_ is the rank of *Y*_*i*,*t*_, *i* = 1, 2, ⋯, *n*, in sample {*X*_1,*t*_, *X*_2,*t*_, ⋯, *X*_*m*,*t*_, *Y*_1,*t*_, *Y*_2,*t*_, ⋯, *Y*_*n*,*t*_} of size *N*( = *m* + *n*). For *m*, *n*⟶+∞ and *m*/*N*⟶ constant *C*. Additionally [68],

(5) $$\begin{array}{c} E\left(\text{M}{\text{D}}_{t}\left|H_{0}\right.\right)=\frac{n\left(N^{2}-1\right)}{12},\\ \text{Var}\left(\text{M}{\text{D}}_{t}\left|H_{0}\right.\right)=\frac{mn\left(N+1\right)\left(N^{2}-4\right)}{180}. \end{array}$$

Filgner and Killeen [69] also introduced a test statistic for scale parameters that is based on the absolute rank. The statistic is defined as

(6) $$\begin{array}{c} F_{t}=\overset{n}{\underset{i=1}{\sum }}R_{i,t}. \end{array}$$

*R*_*i*,*t*_ is the rank of *V*_*i*,*t*_^*R*^ in pooled sample {*V*_1,*t*_^*R*^, *V*_2,*t*_^*R*^, ⋯, *V*_*m*,*t*_^*R*^, *V*_1,*t*_^*T*^, *V*_2,*t*_^*T*^, ⋯, *V*_*n*,*t*_^*T*^}, where *V*_*i*,*t*_^*R*^ = |*X*_*i*,*t*_ − *M*|, *V*_*i*,*t*_^*T*^ = |*Y*_*i*,*t*_ − *M*|. *M* represents the median of the sample {*X*_1,*t*_, *X*_2,*t*_, ⋯, *X*_*m*,*t*_, *Y*_1,*t*_, *Y*_2,*t*_, ⋯, *Y*_*n*,*t*_}. *F*_*t*_ has the distribution of Wilcoxon's rank-sum statistic under the null hypothesis. Therefore,

(7) $$\begin{array}{c} E\left(F_{t}\left|H_{0}\right.\right)=\frac{mn}{2},\\ \text{Var}\left(F_{t}\left|H_{0}\right.\right)=\frac{mn\left(N+1\right)}{12}. \end{array}$$

## 3. Proposed Monitoring Strategy

We assume that there are *m*-independent observations from an unknown multivariate continuous distribution with dimensionality *p*. We assume that independent observations, **X**_**i**_, follow the model below:

(8) $$\begin{array}{c} X_{i}\sim \left\{\begin{array}{c} G_{p}\left(\mu_{0},\Sigma_{0}\right),\;\text{if }i=1,2,\cdots ,\tau ,\\ G_{p}\left(\mu_{1},\Sigma_{1}\right),\;\text{if }i=\tau +1,\tau +2,\cdots , \end{array}\right. \end{array}$$

where *μ*_0_ and *μ*_1_ are the in-control (IC) location vector and the OC location vector, respectively; *Σ*_0_ and *Σ*_1_ represent the IC covariance matrix and the OC covariance matrix, respectively, where (*μ*_0_, *Σ*_0_) ≠ (*μ*_1_, *Σ*_1_); *τ* represents an unknown change point; and **G**_**p**_(·) is an unknown continuous distribution function. In phase I, we assume that the IC sample of size *m* is given at time *t*, *R* = {**X**_1,**t**_, **X**_2,**t**_, ⋯, **X**_**i**,**t**_, ⋯, **X**_**m**,**t**_} where **X**_**i**,**t**_ = {*X*_1,*i*,*t*_, *X*_2,*i*,*t*_, ⋯,*X*_*p*,*i*,*t*_}′, *i* = 1, 2, ⋯, *m*. In phase II, *T* = {**Y**_1,**t**_, **Y**_2,**t**_, ⋯, **Y**_**n**,**t**_} of size *n* is obtained. After the phase I sample *R* is analyzed, the phase II sample *T* is monitored.

Inspired by Mukherjee and Marozzi [50] for multivariate processes, we consider the *p*-dimension statistic of the Euclidean distance of new observations and the mean vector of phase I data, **X**_**i**,**t**_, *i* = 1, 2, ⋯, *m*. That is, $D_{i,t}^{R}=\left\|X_{i,t}-\bar{X}\right\|$ and $D_{i,t}^{T}=\left\|Y_{i,t}-\bar{X}\right\|$, where $\bar{X}=\left(1/m\right)\sum_{i=1}^{m}X_{i,t}$. Now, a univariate phase II sequence is obtained, {*D*_1,*t*_^*R*^, *D*_2,*t*_^*R*^, ⋯, *D*_*m*,*t*_^*R*^, *D*_1,*t*_^*T*^, *D*_2,*t*_^*T*^, ⋯, *D*_*n*,*t*_^*T*^}. Then, a Shewhart-type chart for monitoring location changes that is based on the Wilcoxon rank-sum statistic (i.e., S-W chart) can be constructed. The statistic of the S-W chart is $Z_{W,t}=\left(W_{1,t}-mn/2\right)/\sqrt{mn\left(N+1\right)/12}$ with upper control limit (UCL)

(9) $$\begin{array}{c} \text{UCL}=E\left(Z_{W,t}\left|H_{0}\right.\right)+L\sqrt{\text{Var}\left(Z_{W,t}\left|H_{0}\right.\right)}, \end{array}$$

and lower control limit (LCL)

(10) $$\begin{array}{c} \text{LCL}=E\left(Z_{W,t}\left|H_{0}\right.\right)-L\sqrt{\text{Var}\left(Z_{W,t}\left|H_{0}\right.\right)}, \end{array}$$

where *L* is an unknown constant. The Shewhart-type chart can be constructed based on three other types of hypothesis statistics for the scale parameter. The S-ST chart (i.e., the Shewhart-type chart based on the Siegel-Tukey statistic) is calculated using $Z_{ST,t}=\left(S_{t}-E\left(S_{t}\left|H_{0}\right.\right)\right)/\sqrt{\text{Var}\left(S_{t}\left|H_{0}\right.\right)}$ with $\text{UCL}=E\left(Z_{\text{ST},t}\left|H_{0}\right.\right)+L\sqrt{\text{Var}\left(Z_{\text{ST},t}\left|H_{0}\right.\right)}$ and $\text{LCL}=E\left(Z_{\text{ST},t}\left|H_{0}\right.\right)-L\sqrt{\text{Var}\left(Z_{\text{ST},t}\left|H_{0}\right.\right)}$. The S-MD chart (i.e., the Shewhart-type chart based on the mood statistic) is given as follows: $Z_{\text{MD},t}=\left(\text{M}{\text{D}}_{t}-E\left(\text{M}{\text{D}}_{t}\left|H_{0}\right.\right)\right)/\sqrt{\text{Var}\left(\text{M}{\text{D}}_{t}\left|H_{0}\right.\right)}$ with $\text{UCL}=E\left(Z_{\text{MD},t}\left|H_{0}\right.\right)+L\sqrt{\text{Var}\left(Z_{\text{MD},t}\left|H_{0}\right.\right)}$ and $\text{LCL}=E\left(Z_{\text{MD},t}\left|H_{0}\right.\right)-L\sqrt{\text{Var}\left(Z_{\text{MD},t}\left|H_{0}\right.\right)}$. The S-FK chart (i.e., the Shewhart-type chart based on the Filgner-Killeen statistic) is given by $Z_{\text{FK},t}=\left(F_{t}-E\left(F_{t}\left|H_{0}\right.\right)\right)/\sqrt{\text{Var}\left(F_{t}\left|H_{0}\right.\right)}$ with $\text{UCL}=E\left(Z_{F,t}\left|H_{0}\right.\right)+L\sqrt{\text{Var}\left(Z_{F,t}\left|H_{0}\right.\right)}$, and $\text{LCL}=E\left(Z_{F,t}\left|H_{0}\right.\right)-L\sqrt{\text{Var}\left(Z_{F,t}\left|H_{0}\right.\right)}$.

We then use the average run length (ARL) to evaluate the performance of these methods. ARL is the number of points that, on average, will be plotted on a control chart before an OC condition occurs. If the process is IC, ARL_0_ = 1/*α*; otherwise, ARL_1_ = 1/(1 − *β*) when the process is OC. In addition, *α* is the probability of a type I error occurring, and *β* is the probability of a type II error occurring. Therefore, we typically fix IC ARL, which is denoted as ARL_0_, and compare the OC ARL, which is denoted as ARL_1_. A small ARL_1_ is considered better.  Figure 1 shows the OC ARL of the S-ST, S-MD, and S-FK charts. We let *m* = 50, *n* = {5,10,20}, and *p* = 4 under the multivariate Gaussian distribution with expectations *μ*_0_ and the variance matrix, *Σ*_0_. For a fair comparison, we set ARL_0_ = 500 for all control schemes.  Figure 1 shows the OC ARL of the three Shewhart-type schemes when detecting scale parameters.  Figure 1 shows that the S-MD chart's performance is better than the other charts when detecting a range of scale shifts.

When calculating the Mahalanobis distance, the sample population must exceed the sample dimension; otherwise, the inverse matrix of the population sample covariance matrix obtained does not exist. Thus, the Mahalanobis distance sometimes fails to meet practical requirements. It is also not appropriate to simply use the Euclidean distance to reduce the dimensionality of high-dimensional data, because this process would equate the differences between different data attributes (i.e., the dimensions of each index or variable). The standardized Euclidean distance is an improvement strategy that can overcome the shortcoming of the simple Euclidean distance. Since the distribution of each dimension component of the data is different, the first to “standardize” each component to the associated mean and variance are equal.

Mukherjee and Marozzi [50] consider the sum of the squares of standardized Wilcoxon and Bradley statistics for monitoring high-dimensional processes with unknown parameters. Inspired by Mukherjee and Marozzi [50], we combine the idea of control schemes and hypothesis testing to propose an effective control scheme that simultaneously monitors expectation and variance. Based on this analysis, we propose an alternative control scheme, whose statistic is as follows:

(11) $$\begin{array}{c} Z_{t}=Z_{W,t}+Z_{\text{MD},t}, \end{array}$$

with

(12) $$\begin{array}{c} \text{UCL}=E\left(Z_{t}\left|H_{0}\right.\right)+L\sqrt{\text{Var}\left(Z_{t}\left|H_{0}\right.\right)},\\ \text{LCL}=E\left(Z_{t}\left|H_{0}\right.\right)-L\sqrt{\text{Var}\left(Z_{t}\left|H_{0}\right.\right)}. \end{array}$$

The term asymptotic distribution is used in the sense of convergence in law when *m*⟶∞ and *n*⟶∞ with the ratio *m*/*N* constant [52]. Under *H*_0_, the statistics *Z*_*W*,*t*_ and *Z*_*MD*,*t*_ are uncorrelated for all *m* and *n*. Since, for all *m* and *n*,

(13) $$\begin{array}{c} E\left(W_{2,t}\text{M}{\text{D}}_{t}\left|H_{0}\right.\right)=E\left[\overset{n}{\underset{i=1}{\sum }}{\left(R_{i,t}-\frac{N+1}{2}\right)}^{2}\overset{n}{\underset{j=1}{\sum }}R_{j,t}\left|H_{0}\right.\right],\\ E\left(\overset{n}{\underset{j=1}{\sum }}R_{j,t}\left|H_{0}\right.\right)=\frac{n\left(N+1\right)}{2},\\ E\left(\overset{n}{\underset{i=1}{\sum }}\overset{n}{\underset{j=1}{\sum }}R_{i,t}R_{j,t}\left|H_{0}\right.\right)=\frac{n^{2}\left(N+1\right)\left(3N+2\right)}{12},\\ E\left(\overset{n}{\underset{i=1}{\sum }}\overset{n}{\underset{j=1}{\sum }}R_{i,t}^{2}R_{j,t}\left|H_{0}\right.\right)=\frac{n^{2}N{\left(N+1\right)}^{2}}{6}. \end{array}$$

Thus, we have

(14) $$\begin{array}{c} E\left(W_{2,t}\text{M}{\text{D}}_{t}\left|H_{0}\right.\right)=\frac{n^{2}\left(N-1\right){\left(N+1\right)}^{2}}{24}. \end{array}$$

Equality (14) is the product of *E*(*W*_2,*t*_|*H*_0_) and *E*(MD_*t*_|*H*_0_). Therefore,

(15) $$\begin{array}{c} E\left(W_{1,t}\text{M}{\text{D}}_{t}\left|H_{0}\right.\right)=E\left(W_{1,t}\left|H_{0}\right.\right)E\left(\text{M}{\text{D}}_{t}\left|H_{0}\right.\right). \end{array}$$

It is obvious that

(16) $$\begin{array}{c} E\left(Z_{W,t}Z_{\text{MD},t}\left|H_{0}\right.\right)=E\left(Z_{W,t}\left|H_{0}\right.\right)E\left(Z_{\text{MD},t}\left|H_{0}\right.\right). \end{array}$$

Under *H*_0_, $Z_{W,t}=\left(W_{1,t}-E\left(W_{1,t}\left|H_{0}\right.\right)\right)/\sqrt{\text{Var}\left(W_{1,t}\left|H_{0}\right.\right)}⟶N\left(0,1\right)$ and $Z_{MD,t}=\left(\text{M}{\text{D}}_{t}-E\left(\text{M}{\text{D}}_{t}\left|H_{0}\right.\right)\right)/\sqrt{\text{Var}\left(\text{M}{\text{D}}_{t}\left|H_{0}\right.\right)}⟶N\left(0,1\right)$ with *m*⟶∞, *n*⟶∞, and the ratio *m*/*N* constant.

## 4. Performance Evaluation

In this section, we compare the performances of these charts with different reference sample sizes *m* and test sample sizes *n* when shifts occur. We assume that the *t*th future observation, **X**_**t**_, is collected over time using the following multivariate model:

(17) $$\begin{array}{c} X_{t}\sim \left\{\begin{array}{c} N_{p}\left(\mu_{0},\Sigma_{0}\right),\;\text{for }t=1,2,\cdots ,\tau ,\\ N_{p}\left(\mu_{1},\Sigma_{1}\right),\;\text{for }t=\tau +1,\tau +2,\cdots , \end{array}\right. \end{array}$$

where *μ*_0_ = (0, 0, 0, 0), *μ*_1_ = (0, 0, *δ*, *δ*), and *Σ*_0_ represents the 4 × 4 identity matrix. We let *τ* = 50 and dimensionality *p* = 4.  Table 2 shows the OC ARL of these charts.  Table 3 presents the OC ARL of these charts when there is a correlation between variables:

(18) $$\begin{array}{c} X_{t}\sim \left\{\begin{array}{c} N_{p}\left(\mu_{0},\Sigma_{2}\right),\;\text{for }t=1,2,\cdots ,\tau ,\\ N_{p}\left(\mu_{1},\Sigma_{3}\right),\;\text{for }t=\tau +1,\tau +2,\cdots , \end{array}\right. \end{array}$$

where

(19) $$\begin{array}{c} \Sigma_{2}=\left(\begin{array}{cccc} 1 & 0.2 & 0.2 & 0.2\\ 0.2 & 1 & 0.2 & 0.2\\ 0.2 & 0.2 & 1 & 0.2\\ 0.2 & 0.2 & 0.2 & 1 \end{array}\right),\\ \Sigma_{3}=\left(\begin{array}{cccc} 1+\sigma & 0.2 & 0.2 & 0.2\\ 0.2 & 1 & 0.2 & 0.2\\ 0.2 & 0.2 & 1 & 0.2\\ 0.2 & 0.2 & 0.2 & 1 \end{array}\right). \end{array}$$

The Weibull type of distributional changes for detecting general distributional changes is shown in Table 4, where Weibull(*θ*_1_, *θ*_2_) represents the Weibull distribution with the shape parameter *θ*_1_ and the scale parameter *θ*_2_. The IC distribution is Weibull(1, 1), and the OC distribution is Weibull(1, 1 + *δ*). We also consider the three types of general changes (multivariate *t* with 3 *df*, multivariate exponential, and multivariate gamma distributions) in Table 5. Tables 2–5 show that the proposed method performs well for detecting a range of shifts.

## 5. Illustration

### 5.1. Data Source

To describe the proposed method, we analyze a real clinical case. Samples arrive periodically as Dr. Wolberg reports in his clinical cases. The database therefore reflects this chronological grouping of the data. For each of the 599 clinical cases, several clinical features were observed or measured. Quantitative attributes including clump thickness, uniformity of cell size, uniformity of cell shape, marginal adhesion, single epithelial cell size, bare nuclei, bland chromatin, normal nucleoli, and mitoses. The datasets are publicly available in the “Breast Cancer Wisconsin (Original) Data Set” of the UCI Machine Learning Repository and can be downloaded from the website http://archive.ics.uci.edu/ml/datasets/Breast+Cancer+Wisconsin+%28Original%29. Breast cancer screening is an important strategy to allow for early detection and ensure a greater probability of having a good outcome in treatment. More details about these datasets can be related to [70–73]. In this work, we aim to monitor the Breast Cancer Wisconsin Data Set and identify whether there is a shift in a process.

### 5.2. Data Analysis

A quantile-quantile (Q-Q) plot of each index, including 599 historical observations, is shown in Figure 2, which highlights that the normality assumption is invalid, which leads us to reject the null hypothesis that the data are normally distributed. Thus, we use the proposed distribution-free control scheme to monitor the breast cancer data.

We let *m* = 100 and *n* = 5. We use the 1–350 IC data to find the control limits of the S-W chart, S-MD chart, and proposed chart. For a fair comparison, the IC ARL of all control charts is set equal to 400, and the remaining 249 breast cancer data are monitored. The curves of the S-W and S-MD charts of the monitored banknote authentication data are shown in Figure 3, which indicates that the S-W chart produces a false alarm when the process is IC; conversely, the S-MD chart produces no OC signal when the process is OC.  Figure 4 shows the proposed chart for monitoring breast cancer data and shows that the statistic of the proposed chart falls out of the control limits after 353 observations. Compared with the S-W and S-MD charts, the proposed chart can detect a shift more accurately and earlier than the other charts.

## 6. Conclusions and Discussion

This paper provided a new control scheme for detecting location and scale changes. Inspired by Mukherjee and Marozzi [50], we proposed an effective control chart that simultaneously monitors changes in both location and scale. In this paper, Breast Cancer Wisconsin Data Sets are provided by using the proposed method. Spectral analysis is also reviewed and conducted to investigate the periodicities of shorter time series, and then, nonlinear least squares fitting is used for fitting analysis. The real-data example shows that the proposed scheme performed well for detecting process changes. In this study, we mainly considered the standard Euclidean distance to reduce the dimensionality of high-dimensional data; the other methods of dimensionality reduction still need to be investigated in more detail.

## Figures and Tables

**Figure 1:** Comparison of the three Shewhart-type schemes when detecting changes in scale.

**Figure 2:** Corresponding normal Q-Q plot of the breast cancer data.

**Figure 3:** (a) S-W chart for monitoring breast cancer data. (b) S-MD chart for monitoring breast cancer data.

**Figure 4:** The proposed chart for monitoring breast cancer data.

**Table 1:** Rank of *Q*_(1),*t*_, *Q*_(2),*t*_, ⋯, *Q*_(*m* + *n*),*t*_.

Data	*Q*_(1),*t*_	*Q*_(2),*t*_	*Q*_(3),*t*_	*Q*_(4),*t*_	⋯	*Q*_(*m* + *n* − 3),*t*_	*Q*_(*m* + *n* − 2),*t*_	*Q*_(*m* + *n* − 1),*t*_	*Q*_(*m* + *n*),*t*_
Rank	1	4	5	8	⋯	7	6	3	2

**Table 2:** OC ARL values of these charts for various *m* and *n* when zero-state ARL_0_ = 500 with the IC distribution **N**(*μ*_0_, *Σ*_0_).

*m*	Shifts	S-W	S-MD	Proposed	S-W	S-MD	Proposed	S-W	S-MD	Proposed
50		*n* = 5			*n* = 10			*n* = 20		
	*δ* = 0.5, *σ* = 2	85.5	161.2	69.1	63.7	169.6	48	48.6	251	42.8
	*δ* = 0.5, *σ* = 4	25.1	58.1	16.6	15.1	62.3	11.8	10.8	129.7	9.9
	*δ* = 1, *σ* = 2	26.3	71.7	25.3	16	67.8	15.8	16.9	180.4	16.5
	*δ* = 1, *σ* = 4	9.8	28.9	9.6	6.5	36.1	6.4	5.5	90	5.3

100		*n* = 5			*n* = 20			*n* = 50		
	*δ* = 0.5, *σ* = 2	69.1	12.6	57.6	22.9	110.7	21.2	17.7	180.7	16.2
	*δ* = 0.5, *σ* = 4	16.9	34.4	12.2	5.6	27.8	4.6	4.8	72.1	4.1
	*δ* = 1, *σ* = 2	20.7	42.8	18.5	7.3	40.5	6.9	8	114.8	7.3
	*δ* = 1, *σ* = 4	7.9	14.6	7.5	3.1	11.7	3	2.5	47.4	2.5

200		*n* = 5			*n* = 20			*n* = 50		
	*δ* = 0.5, *σ* = 2	58.3	96.7	49.8	16.7	62.7	14.2	7.8	10.6	7.3
	*δ* = 0.5, *σ* = 4	14.9	23.3	9.8	4.1	15	3.3	2.5	10.6	2.5
	*δ* = 1, *σ* = 2	19	28.3	18.7	4.4	15	4.1	3.5	20.3	3.3
	*δ* = 1, *σ* = 4	6.7	10.5	6.1	2.3	4.3	2.3	2	4.6	2

**Table 3:** OC ARL values of these charts for various *m* and *n* when zero-state ARL_0_ = 500 with the IC distribution **N**(*μ*_0_, *Σ*_2_).

*m*	Shifts	S-W	S-MD	Proposed	S-W	S-MD	Proposed	S-W	S-MD	Proposed
50		*n* = 5			*n* = 10			*n* = 20		
	*δ* = 0.5, *σ* = 2	96	182.6	70.7	63.5	189.9	53.3	53	274	49.9
	*δ* = 0.5, *σ* = 4	24.7	68.4	19.3	15.9	72.7	12.6	11.2	147	10.9
	*δ* = 1, *σ* = 2	31.5	85.7	30.2	19.3	101.5	18.8	19	193.3	18.8
	*δ* = 1, *σ* = 4	11.2	30.8	11	7.1	40.6	6.8	6.1	103.1	6.1

100		*n* = 5			*n* = 20			*n* = 50		
	*δ* = 0.5, *σ* = 2	73	140.9	67.7	23.9	33.2	22.8	22.5	92.2	22.3
	*δ* = 0.5, *σ* = 4	18.4	39.5	14	5.6	33.2	5.1	3.9	92.2	3.7
	*δ* = 1, *σ* = 2	27.8	47	24.1	5.9	13.8	5.8	8.2	143.2	8.2
	*δ* = 1, *σ* = 4	17.7	16.5	22.1	4.8	14.4	4.8	4.5	56.6	4.2

200		*n* = 5			*n* = 20			*n* = 50		
	*δ* = 0.5, *σ* = 2	65.9	120.3	57.9	16.2	79	16.2	8.8	77.8	8.4
	*δ* = 0.5, *σ* = 4	15.5	27.8	11.3	4	12.2	3.4	2.5	13.4	2.5
	*δ* = 1, *σ* = 2	18.9	34.8	17.6	4.7	16.6	4.3	2.9	23.8	2.7
	*δ* = 1, *σ* = 4	7.5	12.6	7.5	2.4	4.7	2.4	2	5.5	2

**Table 4:** OC ARL values of these charts for various *m* and *n* when zero-state ARL_0_ = 500 with the IC distribution Weibull(1, 1).

*m*	*δ*	S-W	S-MD	Proposed	S-W	S-MD	Proposed	S-W	S-MD	Proposed
50		*n* = 5			*n* = 10			*n* = 20		
	2	5.5	10.3	4	3.7	6.3	2.8	2.6	5.2	2.3
	4	2.3	2.5	2	2.1	2.1	2	2	2.1	2
	6	2.1	2.1	2	2	2	2	2	2	2

100		*n* = 5			*n* = 20			*n* = 50		
	2	5	7.2	3.8	2.3	2.8	2.1	2	2.4	2
	4	2.2	2.2	2	2	2	2	2	2	2
	6	2	2	2	2	2	2	2	2	2

200		*n* = 5			*n* = 20			*n* = 50		
	2	4.6	5.8	3.4	2.2	2.3	2.2	2	2	2
	4	2.2	2.1	2	2	2	2	2	2	2
	6	2	2	2	2	2	2	2	2	2

**Table 5:** OC ARL values of these charts for various *n* when *m* = 100 and zero-state ARL_0_ = 500 under other types of distribution.

*τ*	Type	S-W	S-MD	Proposed	S-W	S-MD	Proposed	S-W	S-MD	Proposed
50		*n* = 5			*n* = 20			*n* = 50		
	1	43.1	126.1	37.5	10.2	103.2	9.4	4.5	252.1	6.9
	2	13.3	64.4	8.1	4.7	5.5	2.8	3.6	10.7	2.4
	3	11.8	59	7.7	4.7	5.5	2.8	3.5	10.3	2.4

100		*n* = 5			*n* = 20			*n* = 50		
	1	43	129.6	41.1	10.1	104.8	9.42	4.4	238.9	6.7
	2	12.7	65.4	7.7	4.8	5.8	2.7	3.4	10.5	2.4
	3	12.5	54.5	7.9	4.6	5.6	2.7	3.6	10.4	2.4

200		*n* = 5			*n* = 20			*n* = 50		
	1	42.9	132.9	39.1	10.7	109.7	9.2	4.7	243.3	6.9
	2	13.4	61.5	8.1	4.8	5.7	2.8	3.4	10.2	2.3
	3	12	58.8	8	4.7	5.7	2.8	3.5	10.6	2.4

1: multivariate *t* with 3 *df* distribution; 2: multivariate gamma distribution; 3: multivariate exponential distribution.

## Data Availability

The data used to support the findings of this study are available from the corresponding author upon request.
